RETRACTED

# Allopregnanolone restores the tyrosine hydroxylase‐positive neurons and motor performance in a 6‐OHDA‐injected mouse model

**DOI:** 10.1111/cns.13432

**Published:** 2020-06-30

**Authors:** Zhi‐Chi Chen, Tong‐Tong Wang, Wei Bian, Xin Ye, Meng‐Yi Li, Juan‐Juan Du, Peng Zhou, Huai‐Rui Cui, Yu‐Qiang Ding, Yan‐hua Ren, Shuang‐Shuang Qi, Yuan‐Yuan Yuan, Min Liao, Chen‐You Sun

**Affiliations:** ^1^ Department of Anatomy School of Basic Medical Sciences Wenzhou Medical University Wenzhou China; ^2^ Institute of Neuroscience School of Basic Medical Sciences Wenzhou Medical University Wenzhou China; ^3^ Department of Histology and Embryology School of Basic Medical Sciences Wenzhou Medical University Wenzhou China; ^4^ Department of Pharmacy Second Affiliated Hospital Wenzhou Medical University Wenzhou China; ^5^ School of Basic Medical Sciences Zhejiang Chinese Medical University Hangzhou China

**Keywords:** 6‐hydroxydopamine, allopregnanolone, brain‐derived neurotrophic factor, calcium/calmodulin‐dependent protein kinase II delta 3, neural progenitor cell, γ‐aminobutyric acid A receptor

## Abstract

**Aims:**

It has been reported that allopregnanolone (APα) promotes the neurogenesis of the neural progenitor cells (NPCs) in the subventricular zone (SVZ) and prevents the decrease of dopaminergic neurons in 6‐hydroxydopamine (6‐OHDA)‐treated mice by binding to γ‐aminobutyric acid A receptor (GABAAR) and then opening voltage‐gated L‐type Ca^2+^ channel, but the underlying mechanisms remain elusive. The aim of this study was to explore the possible involvement of GABAAR and calcium/calmodulin‐dependent protein kinase II delta 3 (CaMKIIδ3) in this process.

**Methods:**

6‐OHDA‐treated mice and primary cultured midbrain cells were administrated with APα and GABAAR antagonist bicuculline (Bic), and the proliferation and differentiation of NPCs, the tyrosine hydroxylase (TH)‐positive neurons and their fibers, the expression levels of CaMKIIδ3 and brain‐derived neurotrophic factor (BDNF), and motor functions were measured using ELISA, immunohistochemical staining, real‐time RT‐PCR, Western blot, and behavioral test.

**Results:**

Allopregnanolone significantly promoted the phosphorylation of cytoplasmic CaMKIIδ3 and its nuclear translocation by binding to GABAAR, which, in turn, increased the expression levels of BDNF. This may account for the findings that the exogenous APα enhanced the proliferation and differentiation of NPCs, and ameliorated the nigrostriatal system and behavioral performance in 6‐OHDA‐treated mice.

**Conclusions:**

Allopregnanolone may directly activate GABAAR, which, in turn, enhance the proliferation and differentiation of NPCs *via* upregulating the expression levels of CaMKIIδ3, and finally contribute to the restoration of dopaminergic neurons in 6‐OHDA‐treated mice.

RETRACTED

## Graphical abstract

APα significantly promotes the phosphorylation of cytoplasmic CaMKIIδ3 and its nuclear translocation by binding to GABAAR, which, in turn, increases the expression levels of cell cycle protein and BDNF. This may account for the findings that APα enhances the proliferation and differentiation of NPCs, and ameliorates the deficiency of dopaminergic neurons in 6‐OHDA‐treated mice and primary cultured midbrain cells.

## 1 INTRODUCTION

Parkinson's disease (PD) is characterized by the reduction of dopaminergic neurons in the substantia nigra (SN) and the subsequent dopamine depletion in the striatum.^1^ The resting tremor, movement slowness, and postural instability have become the most common clinical symptoms of PD.^2^, ^3^ 6‐hydroxydopamine (6‐OHDA) and 1‐methyl‐4‐phenyl‐1, 2, 3, 6‐tetrahydropyridine (MPTP) are commonly used to develop PD animal models.^4^, ^5^ Some studies reported that the generation of stem cells in the subventricular zone (SVZ) lining the lateral ventricles (LVs) was inhibited in the rats or mice treated with 6‐OHDA or MPTP.^6^, ^7^ Another study suggested that the neurodegeneration might result from the disturbance between the neurogenesis and neuronal cell loss.^8^ Our previous study found that 6‐OHDA‐treated mice had an incomplete recovery of dopaminergic neurons in SN, suggesting that a potential therapeutic approach to promote the neurogenesis should be developed in PD treatment.^9^, ^10^

Allopregnanolone (APα), which is synthesized in the embryonic and adult central nervous system (CNS), as well as in the neural progenitor cells (NPCs), shows a neurodegenerative disease‐associated decline.^11^, ^12^, ^13^ In Alzheimer's disease (AD) mice, some reports have indicated that APα promotes the proliferation of NPCs in the LV‐SVZ, and prevents the reduction of tyrosine hydroxylase (TH)‐expressed neurons in SN pars compacta (SNpc).^8^, ^10^, ^14^, ^15^, ^16^ In addition, Adeosun et al^17^ reported that APα ameliorated the deficits of motor function in MPTP‐injected mice. However, the mechanisms underlying APα‐involved neuroprotective effects remain unknown.

Accumulated evidences have indicated that APα increases an efflux of chloride through the depolarization of γ‐aminobutyric acid A receptor (GABAAR)‐driven opening of voltage‐gated L‐type Ca^2+^ channel (VGLCC), and the elevated Ca^2+^ signaling might activate the calcium/calmodulin (CaM)‐dependent protein kinase II (CaMKII) in immature neurons.^14^, ^18^, ^19^ As a multifunctional serine/threonine protein kinase, CaMKII plays an important biological role in a variety of cellular processes.^20^ CaMKII subunits including α, β, γ, and δ have been identified, and among them CaMKII delta 3 (CaMKIIδ3) is highly expressed in the dopaminergic neurons of SN.^21^ The nuclear CaMKII can regulate the transcription of brain‐derived neurotrophic factor (BDNF), and BDNF, in turn, promotes the neuronal survival and the growth of axon and dendrites.^20^, ^21^ It is likely that APα‐induced proliferation and differentiation of NPCs might depend on CaMKIIδ3 and BDNF, in which APα might regulate the activity of GABAAR.

RETRACTED

In this study, 6‐OHDA‐treated mice and primary cultured midbrain cells were administrated with APα and/or bicuculline (Bic, a specific blocker of GABAAR) to evaluate the effects of APα and its possible molecular mechanism.

## 2 MATERIALS AND METHODS

### 2.1 Animals

All experiments should comply with National Institute of Health Guide for Care and Use of Laboratory Animals (NIH Publications No. 8023, revised 1978) and Animal Committee of Wenzhou Medical University. In order to identify SVZ‐derived NPCs and explore their proliferation, *Nestin‐CreER^TM^::ROSA26‐LacZ* mice was used.^9^ Tamoxifen (TAM, Sigma; T5648) that was predissolved in the corn oil (15 mg/mL; vehicle solution) can activate *Cre* to excise the transcriptional stop cassette flanked by *LoxP* sites in *ROSA‐LacZ* reporter mice and induce the expression of *LacZ* gene in NPCs. β‐galactosidase (β‐gal) that was encoded by *LacZ* gene could catalyze the hydrolysis of lactose and the hydrolysate showed as blue color by X‐gal staining. Thus, X‐gal‐stained cells were regarded as Nestin‐positive NPCs. *Nestin‐CreER^TM^*::*ROSA‐LacZ* mice were intraperitoneally (i.p.) injected with TAM (200 ~ 250 mg/kg/d) or the same amount of vehicle solution for five consecutive days.

A total of 3‐month‐old adult male *Nestin‐CreER^TM^::ROSA26‐LacZ* mice (n = 48) and wild‐type C57BL/6 (n = 48) were maintained at a 12‐hour light/dark cycle, temperature/humidity‐controlled animal facility with free access to food and water. These mice were randomly assigned to normal saline + DMSO, normal saline + APα, normal saline + Bic, 6‐OHDA + DMSO, 6‐OHDA + APα, and 6‐OHDA + APα+Bic groups. In order to develop PD mouse model, 6‐OHDA (Sigma; H4381) that was predissolved in 0.02% L‐ascorbate normal saline (10.26 μg/μL) was used to obtain the degeneration of dopaminergic neurons. The right side of striatum was stereotaxically given 6‐OHDA by a double point administration in each point having 0.487 μL according to anterior‐posterior (−2.0 and −2.3 mm), medial‐lateral (1.0 and 0.3 mm), and dorsal‐ventral (−3.5 mm) with respect to bregma using a 5‐μl Hamilton syringe. In the previous studies, we found that a single 20 mg/kg of APα injection could significantly alleviate the deficiency of TH‐positive neurons in AD‐transgenic mouse model^8^, ^10^; thus in this study, 20 mg/kg of APα (Tocris Bioscience; 3653) was subcutaneously given once on day 7 after 6‐OHDA injection. In order to explore the alteration that APα exerted the neurogenic effects when the function of GABAAR was blocked by Bic, 4 mg/kg of Bic (Tocris Bioscience; 48954) was given (i.p.) to obtain an IC50 of 2 ~ 3 µmol/L at 0.5 hour prior to APα injection.^22^, ^23^ In order to analyze the cell proliferation, 100 mg/kg of bromodeoxyuridine (BrdU, Sigma; B5002) was (i.p.) injected once daily for four consecutive days at 1 hour prior to 6‐OHDA or APα or Bic or vehicle solution administrations. Mice were sacrificed at 2, 4, and 6 weeks following 6‐OHDA for 6‐OHDA + DMSO or 7, 21, and 35 days following APα or Bic administrations for 6‐OHDA + APα and 6‐OHDA + APα+Bic groups.

RETRACTED

### 2.2 Primary culture of midbrain cells

The fetuses of pregnant SD rats were obtained on embryonic day 12. The ventral part of midbrain was dissociated into cells and maintained in 500 μL of serum‐free Neurobasal medium/B27 supplement (Gibco Invitrogen; 21103049/17504044) at 37°C and 5% CO2 atmosphere. On the first day in vitro (DIV 1), these midbrain‐derived cells were incubated with the mouse anti‐Nestin antibody (1:400; Cell Signaling Technology; 33475S) to identify the neurospheres. Thereafter, these cells were divided into the control, normal saline + DMSO, normal saline + APα, normal saline + Bic, and 6‐OHDA‐treated groups in combination with either DMSO or 5, 50, 500 nmol/L, and 1 μmol/L concentrations of APα. The cells treated without any chemicals and reagents were used as the control group. Once the most optimal APα concentration was determined, these cells were further divided into 6‐OHDA‐treated group administrated with APα and/or Bic on DIV 3. In 6‐OHDA + APα+Bic group, the cells were pretreated with 30 μmol/L Bic at 30 minutes prior to APα administration and then cultured for 24 hours before 0.1 mmol/L 6‐OHDA was given for 24 hours. In addition, each group of cells was exposed to 10 μmol/L BrdU at 1 hour prior to 6‐OHDA or APα or Bic or vehicle solution treatment.

### 2.3 Behavioral test

One day prior to sacrifice, the behavioral tests were performed in sequences with a 30‐minute interval.

#### 2.3.1 Apomorphine‐induced turning behavior

Mice were injected (i.p.) with apomorphine (Sigma; 41372‐20‐7) at a dose of 0.125 g/L and then placed into a measuring cup to record the circles that the mice rotated toward a non‐6‐OHDA‐injected side within 20 minutes. The apomorphine‐induced turnings were expressed as circles/min.

RETRACTED

#### 2.3.2 Open‐field test

Each mouse was placed at the center of a 25‐square floor (16 × 16 cm/square) in a box and then practiced a 5‐minute session (pretest) for habituation to the new environment. On day 1 following the pretest session, the mice were allowed to explore for 5 minutes, and the total walking distance (mm) and an average walking velocity (mm/s) were recorded within 5 minutes.^22^, ^23^

#### 2.3.3 Rotarod test

Mice were successively placed onto a still and moving rod for 2 ~ 3 minutes. The speed of rod was progressively increased to 60 rpm until the mice fell off the rotating rod. The time latency (sec) and the velocity (r/min) of rotating rod were recorded before or when the mice fell off the rotating rod.

### 2.4 Quantification of APα and dopamine

In order to determine the effect of exogenous APα on the endogenous APα and dopamine in 6‐OHDA‐injected mice, APα or dopamine concentration in the cerebral cortex or striatum was measured by comparing the optical densities (OD) of samples to the standard curve according to the manufacturer's instruction of ELISA kit (Lab‐bio Biomart). Briefly, fifty microliters of blank control, APα, or dopamine standard and tissue samples was placed into a 96‐well plate that was precoated with the monoclonal anti‐APα or dopamine antibody. Afterward, fifty microliters of biotin‐conjugated polyclonal antibody was added and incubated for 45 minutes at 37°C. Finally, one hundred microliters of avidin‐conjugated horseradish peroxidase (HRP) was added, followed by an incubation with 90 µL chromogen solution for 15 minutes at 37℃. Having added 50 µL stopping solution, the color change was assayed at 450‐nm wave length using a microplate absorbance reader (Elx800, BioTek).

### 2.5 X‐gal and immunofluorescent staining

The staining of X‐gal and immunofluorescence was performed, as reported previously with slight modifications.^8^, ^9^, ^10^ Briefly, six sets of sequential coronary sections (40‐μm thickness) were collected. The brain sections were subjected to X‐gal staining solution (Sigma; BG‐3) overnight and then counterstained with 0.1% neutral red (Sigma; N4638) for 1 hour at 37°C. To analyze the proliferation and differentiation of cultured midbrain NPCs, each group of cells was incubated overnight with the rabbit anti‐doublecortin (DCX; 1:400; Cell Signaling Technology; 148025) on DIV 5, or rabbit anti‐β‐tubulin III (1:400; Cell Signaling Technology; 151155) on DIV 7, or guinea pig anti‐neuronal nuclear antigen (NeuN; 1:3000; Merck Millipore; ABN90) on DIV 15, or rabbit anti‐TH antibodies (1:400; Merck Millipore; AB152) on DIV16 alone or in combination with the mouse anti‐BrdU antibody (1:400; Novus; NB500‐169). The cells were then incubated with DyLight594 goat anti‐mouse or DyLight488 goat anti‐rabbit secondary antibody (1:400; Jackson ImmunoResearch) for 1.5 hours at 37°C. Finally, the cells were cover‐slipped with DAPI‐containing mounting medium (Sigma). Negative control was carried out by replacing with normal serum or vehicle solution.

RETRACTED

### 2.6 Immunostaining for TH‐positive fibers

The brain sections were incubated with the rabbit anti‐TH antibody (1:400; Merck Millipore; AB152) overnight at 4°C and then incubated with the goat anti‐rabbit secondary antibody (1:400; Jackson ImmunoResearch) for 2.5 hours. Finally, TH immunoreactivity was visualized by an incubation of brain sections with 0.05% diaminobenzidine (DAB; Sigma) and 0.01% H2O2 for 5 minutes.

### 2.7 Real‐time RT‐PCR

The total RNA was prepared using TRIzol Reagent (Thermo Fisher Scientific), and the relative expressions of CaMKIIδ3, BDNF, and CDC2 mRNAs were quantified using 2‐ΔΔCT method by qPCR Master Mix reagent (Thermo Fisher Scientific). The mRNA expression of each sample was expressed as the percentage of normal saline + DMSO group.

### 2.8 Western blot

The cytoplasmic and nuclear fractions were extracted according to the manufacturer's instruction (Beyotime). Briefly, the midbrain (~10 mg) was homogenized by sonication with 50 μL lysis buffer containing phenylmethanesulfonyl fluoride (PMSF) and phosphatase inhibitors. The lysate of brain tissue was centrifuged at 9676.8 *g* for 5 minutes at 4°C. The supernatant was transferred to a prechilled 1.5 mL tube (cytoplasmic protein fraction). Fifty microliters of nuclear extraction buffer was added to the tube loading the precipitation, vibrated vigorously for 30 seconds, and then incubated on ice for 2 minutes. The tube was centrifuged at 11 708.9 *g* for 10 minutes at 4°C, and the supernatant was transferred to a prechilled 1.5 mL tube (nuclear protein fraction).

Forty micrograms of protein that was isolated from the midbrain was run onto 10% polyacrylamide gel for 1.5 hours at 80 V and then electro‐transferred onto a polyvinylidene fluoride (PVDF) membrane for 1 hour at 320 mA. The nonspecific binding sites were blocked with 5% nonfat milk for 2 hours. The membrane was incubated overnight at 4°C with the following primary antibodies: rabbit anti‐CaMKIIδ3 or p‐CaMKIIδ3 (T286) or CDK1 or p‐CDC2 (T14) (1:1000; Abcam; ab181052; ab171095; ab32384) or BDNF (1:3000; Merck Millipore; MABN79) or mouse anti‐β‐actin (1:2000; Abgent; AM1829b) or rabbit anti‐Histone H3 (1:1000; Abcam; ab791) antibody. The membrane was then incubated with the corresponding HRP‐conjugated goat anti‐rabbit/mouse antibody (1:5000; ZSGBBIO) for 2 hours at room temperature. The immunoreactivity of protein band was detected with an enhanced chemiluminescent (ECL) kit (Beyotime). The protein level was normalized with respect to β‐actin or Histone H3 (a loading control).

RETRACTED

### 2.9 Co‐immunoprecipitation assay

According to the manufacturer's instruction (Absin), 10% cytoplasmic or nuclear fraction from the midbrain was taken out as an input (positive control). Meanwhile, the remaining extract was coated with 1 ~ 5 μg of rabbit anti‐CaMKIIδ3 or p‐CaMKIIδ3 antibody (Abcam) or IgG (negative control) overnight at 4°C. The extract was then incubated with Protein A and G Sepharose beads (1:1) for 3 hours at 4°C. The magnetic beads were washed thoroughly for 3 times. The input and immunoprecipitation were undertaken by Western blot analysis for CDK1 or BDNF.

### 2.10 Image acquisition, cell counting, and statistical analysis

According to the atlas of mouse brain,^24^ every sixth brain section was collected. An unbiased stereological estimation was made in TH‐positive neurons and X‐gal‐positive cells from 16 randomly selected frames.^9^ In the primarily cultured midbrain cells, the immunopositive cells were counted by randomly selecting five visual fields. In order to measure the OD of striatal TH‐positive fibers, five brain sections were obtained. The immunoreactivity and immunopositive cells were captured under an upright microscope (Olympus) and calculated using ImageJ software (NIH). To identify the colocalization of double‐positive cells, the confocal laser scanning microscope (NIKON A1R) was used to make a 3D (*x‐y, x‐z,* and *y‐z*) reconstruction. Statistical analysis was displayed with Prism 7.04 software (GraphPad Software Inc). All data were presented as mean ± SEM and analyzed by repeated measures of *one‐way* ANOVA or *two‐way* ANOVA followed by Bonferroni post hoc test. The differences were statistically significant when the probability (*P*) value was less than or equal to .05, .01, .001, and .0001.

## 3 RESULTS

### 3.1 APα ameliorated the deficits of balance and coordination in 6‐OHDA‐administrated mice

The open‐field and rotarod tests, as well as the rotational behavior, which mirrored the abilities of balance and coordination, were conducted. 6‐OHDA‐administrated mice displayed a stronger turning behavior toward a noninjected side in response to the apomorphine, as well as a much worse behavioral performance in the open‐field and rotarod tests, as compared with the pretest, and normal saline + DMSO‐ or normal saline + APα‐ or normal saline + Bic‐treated mice. There was not significantly different among the pretest, normal saline + DMSO‐, normal saline + APα‐, and normal saline + Bic‐treated mice. Moreover, the turning behavior was significantly alleviated at 6 weeks, as compared with that at 2 week following 6‐OHDA injection. APα ameliorated the rotational behavior, and reversed the behavioral deficits of 6‐OHDA‐lesioned mice in the open‐field and rotarod tests. Notably, the rotational circles were much less on day 21 and 35 following APα administration. Importantly, APα‐induced behavioral amelioration was blocked by Bic administration (Figure 1A ~ E).

**Figure 1:** (A)~(E), Rotational circles (A), total walking distances (B) and average walking velocity (C) of the open filed test, as well as the time latency (D) and the velocity of rotating rod (E) before or when falling off the rotarod test. Values are mean ± SEM; n = 6~10 at various time points for each group. (F)~(G), Dopamine or APα content in the striatum (F), or cerebral cortex (G). Values are mean ± SEM; n = 2~3 at various time points for each group. **P ＜ .01, ***P ＜ .001, and ****P ＜ .0001, comparison between 6‐OHDA + DMSO and the pretest or normal saline + DMSO or normal saline + APα or normal saline + Bic groups; ^#^ *P ＜ *.05, ^##^ *P ＜ *.01, ^###^ *P ＜ *.001, and ^####^ *P ＜ *.0001, comparison between 6‐OHDA + APα and 6‐OHDA + DMSO groups; ^&^ *P ＜ *.05 and ^&&&&^ *P ＜ *.0001, comparison between 6‐OHDA + APα+Bic and 6‐OHDA + APα groups; ^$^ *P ＜ *.05, ^$$^ *P ＜ *.01, and ^$$$$^ *P ＜ *.0001, comparison between at 2 and 4 or 6 wk following 6‐OHDA injection in the rotational behavior and dopamine or APα content; ^^^^^^ *P ＜ *.0001, comparison between on day 7 and 21 or 35 following APα injection in the rotational behavior or dopamine content using *two‐way* ANOVA followed by Bonferroni post hoc test. NS, no significance

RETRACTED

### 3.2 APα reversed the striatal dopamine level in 6‐OHDA‐injected mice

Since SN dopaminergic neurons projected their axon terminals into the striatum, we examined the striatal dopamine level. There was a significant reduction in the striatal dopamine level of 6‐OHDA + DMSO group, as compared with normal saline + DMSO, normal saline + APα, and normal saline + Bic‐treated groups. There was not significantly different among the normal saline + DMSO‐, normal saline + APα‐, and normal saline + Bic‐treated mice. Moreover, the striatal dopamine level was much higher at 6 weeks than that at 2 weeks following 6‐OHDA injection (*P = *.0041). APα significantly increased the striatal dopamine level of 6‐OHDA + DMSO group, and in particular, there was a striatal dopamine turnover on day 21 and 35 following APα administration (*P = *.0015). It should be noted that these effects were blocked by Bic treatment (Figure 1F).

RETRACTED

### 3.3 Bic blocked the elevation of APα level in the cerebral cortex of 6‐OHDA‐injected mice

In the CNS, APα was mainly synthesized in the cerebral cortex of adult mammal animals,^8^ so we examined APα concentration in the cerebral cortex. There was a significant reduction in APα content of 6‐OHDA + DMSO group at 2 and 4 weeks following 6‐OHDA injection, as compared with normal saline + DMSO‐, normal saline + APα‐, and normal saline + Bic‐treated groups. When the exogenous APα was injected to 6‐OHDA‐treated mice, an increase in APα content occurred on day 7 and 21 following APα injection (*P = *.0063), and this change was blocked again by Bic treatment. However, there did not exist a significant difference among groups at 6 weeks following 6‐OHDA injection (Figure 1G).

### 3.4 Administered APα protected the nigrostriatal system against 6‐OHDA lesion

6‐OHDA was stereotaxically injected into the striatum to induce the lesion of nigrostriatal system. The dopaminergic neurons and their fibers were immunostained with anti‐TH (rate‐limiting enzyme for dopamine biosynthesis) antibody.^25^ TH‐positive neurons in the SN exhibited green immunofluorescence in the perikarya and proximal dendrites (Figure 2A ~ F), and TH‐positive fibers in the striatum displayed brown reaction products (Figure 2G ~ L).

**Figure 2:** (A)~(F), TH‐immunofluorescent stained positive neurons were observed in the SNpc of normal saline + DMSO (A), normal saline + APα (B), normal saline + Bic (C), 6‐OHDA + DMSO (D), 6‐OHDA + APα (E), and 6‐OHDA + APα+Bic (F). (G)~(L), DAB‐stained TH‐positive fibers were observed in the striatum of normal saline + DMSO (G), normal saline + APα (H), normal saline + Bic (I), 6‐OHDA + DMSO (J), 6‐OHDA + APα (K), and 6‐OHDA + APα+Bic (L). SNpc, pars compacta of substantia nigra; VTA, ventral tegmental area; CPu, striatum. Scale bar = 200 μm for images (A)~(L). (M) and (N), Absolute number of TH‐positive neurons in the SNpc (M) and the OD of TH‐positive fibers in the striatum (N) at 2, 4, and 6 wk following 6‐OHDA injection. Values are mean ± SEM; n = 3 at various time points for each group. ****P ＜ .0001, comparison between 6‐OHDA + DMSO and normal saline + DMSO or normal saline + APα or normal saline + Bic groups; ^##^ *P ＜ *.01, ^###^ *P ＜ *.001, and ^####^ *P ＜ *.0001, comparison between 6‐OHDA + APα and 6‐OHDA + DMSO groups; ^&&^ *P ＜ *.01, ^&&&^ *P ＜ *.001, and ^&&&&^ *P ＜ *.0001, comparison between 6‐OHDA + APα+Bic and 6‐OHDA + APα groups; ^$^ *P ＜ *.05, comparison between at 2 and 6 wk following 6‐OHDA injection in the striatal TH‐positive fibers; ^^^^ *P ＜ *.01 and ^^^^^^ *P ＜ *.0001, comparison between on day 7 and 21 or 35 following APα injection in SNpc TH‐positive neurons using *Two‐way* ANOVA followed by Bonferroni post hoc test. NS, no significance

The mice treated with 6‐OHDA had an approximate 71.9%, 58.9%, and 58.05% loss in SNpc TH‐positive neurons, as well as 70.50%, 65.50%, and 57.53% reduction in striatal TH‐positive fibers at 2, 4, and 6 weeks following 6‐OHDA injection, as compared with normal saline + DMSO. There was not significantly different among the normal saline + DMSO‐, normal saline + APα‐, and normal saline + Bic‐treated mice. Moreover, a slight recovery in TH‐positive axon terminals began at 6 weeks following 6‐OHDA injection (*P = *.0208). APα significantly augmented the number of SNpc TH‐positive neurons and OD of their striatal fibers of 6‐OHDA + DMSO group, and in particular, there was a significant increase in TH‐positive neurons on day 21 and 35 following APα administration (*P = *.0163, *P = *.0021). In addition, Bic significantly reduced SNpc TH‐positive neurons and striatal TH immunoreactivity after APα treatment (Figure 2M ~ N).

RETRACTED

### 3.5 APα administration further increased the number of Nestin‐positive NPCs in 6‐OHDA‐injected mice

Our findings showed that X‐gal‐labeled Nestin‐positive NPCs with blue products were prevalent in the SVZ of LV (LV‐SVZ), third ventricle (3V‐SVZ), and cerebral aqueduct (Aq‐SVZ) (Figure 3A ~ C). Relative to normal saline + DMSO group, the ratio of NPCs at 2, 4, and 6 weeks following 6‐OHDA injection was 391.67%, 553.85%, and 156.25% in LV‐SVZ, 298.46%, 800.00%, and 106.25% in 3V‐SVZ, as well as 122.32%, 687.50%, and 286.67% in Aq‐SVZ, respectively. Thus, a peak increase in Nestin‐positive NPCs of these SVZ occurred at 4 weeks following 6‐OHDA injection. There was not significantly different among the normal saline + DMSO‐, normal saline + APα‐, and normal saline + Bic‐treated mice. APα further increased the number of Nestin‐positive NPCs in these SVZ, particularly at 4 weeks following 6‐OHDA injection. In addition, Bic partly abolished APα‐induced increase in NPCs of SVZ (Figure 3D ~ F).

**Figure 3:** (A)~(C), The blue color of X‐gal‐labeled Nestin‐positive NPCs indicated with black arrows were mainly located in the SVZ of LV (A), 3V (B), and Aq (C). LV, lateral ventricle; 3V, the third ventricle; Aq, cerebral aqueduct. Scale bar = 200 μm for images (A)~(C). (D)~(F), Quantification of the ratio of X‐gal‐labeled Nestin‐positive NPCs relative to normal saline + DMSO group in the SVZ of LV (D), 3V (E), and Aq (F) at 2, 4, and 6 wk following 6‐OHDA injection among groups. Values are mean ± SEM; n = 3 at various time points for each group. ****P ＜ .0001, comparison between 6‐OHDA + DMSO and normal saline + DMSO or normal saline + APα or normal saline + Bic groups; ^##^ *P ＜ *.01, ^###^ *P ＜ *.001, and ^####^ *P ＜ *.0001, comparison between 6‐OHDA + APα and 6‐OHDA + DMSO groups; ^&&^ *P ＜ *.01, ^&&&^ *P ＜ *.001, and ^&&&&^ *P ＜ *.0001, comparison between 6‐OHDA + APα+Bic and 6‐OHDA + APα groups; ^$$$$^ *P ＜ *.0001, comparison between at 4 and 2 or 6 wk following 6‐OHDA injection; ^^^^^^ *P ＜ *.0001, comparison between on day 21 and 7 or 35 following APα administration using *two‐way* ANOVA followed by Bonferroni post hoc test. NS, no significance

RETRACTED

### 3.6 APα administration promoted the proliferation and differentiation of 6‐OHDA‐treated midbrain‐derived NPCs

To explore the effects of APα on the NPCs of midbrain, the embryonic midbrain‐derived cells were cultured. A majority of cultured midbrain cells could form neurospheres on DIV 1 (Figure 4A). After these cells were exposed to BrdU for 48 hours, BrdU‐positive cells exhibited a medium‐sized round or oval nucleus, which resembled a chromatin‐like structure (Figure 4B ~ E). BrdU‐labeled newborn midbrain‐derived cells were dramatically decreased in 6‐OHDA‐treated group, as compared with the control group, normal saline + DMSO, normal saline + APα, and normal saline + Bic groups. A series of concentrations of APα (5 nmol/L ~ 1 μmol/L) significantly increased the number of newborn midbrain‐derived cells. Moreover, 500 nmol/L APα was selected as the most optimal APα concentration in promoting the proliferation of these newborn midbrain‐derived cells (data not shown).

**Figure 4:** (A)~(E), Neural stem cells (A), immature NPCs (B), developing neurons (C), mature neurons (D) and dopaminergic neurons (E) were detected using anti‐Nestin, DCX, β‐tubulin III, NeuN, and TH antibodies on DIV 1, 5, 7, 15, and 16, respectively. A representative image of DCX, β‐tubulin III, NeuN and TH‐positive cells (green color), and BrdU‐positive cells (red color) was shown to verify their colocalization in three planes (*x*, *y*, and *z*) by confocal laser scanning microscope. Scale bar = 200, 50, and 100 μm for images (A), (B) and (C)~(E). (F)~(I), The number of DCX, BrdU or DCX/BrdU (F), β‐tubulin III, BrdU or β‐tubulin III/BrdU (G), NeuN, BrdU or NeuN/BrdU (H), and TH, BrdU or TH/BrdU‐positive cells (I) was calculated per field among different groups. Values are mean ± SEM; n = 3 at various time points for each group. **P ＜ .01, ***P ＜ .001, and ****P ＜ .0001, comparison between 6‐OHDA + DMSO and control group or normal saline + DMSO or normal saline + 500 nmol/L APα or normal saline + Bic groups; ^#^ *P ＜ *.05, ^##^ *P ＜ *.01, ^###^ *P ＜ *.001, and ^####^ *P ＜ *.0001, comparison between 6‐OHDA + 500 nmol/L APα and 6‐OHDA + DMSO groups; ^&^ *P ＜ *.05, ^&&^ *P ＜ *.01, and ^&&&&^ *P ＜ *.0001, comparison between 6‐OHDA + 500 nmol/L APα + Bic and 6‐OHDA + 500 nmol/L APα groups by repeated measures of *one‐way* ANOVA followed by Bonferroni post hoc test. NS, no significance

To further investigate the differentiation of midbrain‐derived BrdU‐positive newborn cells, we performed a double immunofluorescence staining. DCX‐positive immature NPCs exhibited a clustermorphology, β‐tubulin III‐positive cells showed a prominent nucleus and neurite extension, NeuN was localized within the nuclear fraction, and TH was mainly present in the cytoplasm (Figure 4B ~ E). After an incubation with BrdU for 48 hours, BrdU‐positive cells were coexpressed with DCX (43.8831 ± 4.5595%) on DIV 5, β‐tubulin III (49.1615 ± 2.4661%) on DIV 7, NeuN (1.8316 ± 0.8350%) on DIV 15, and TH (2.5895 ± 0.0570%) on DIV 16 in the control group. 6‐OHDA significantly caused a decrease in the number of DCX and DCX/BrdU, β‐tubulin III and β‐tubulin III/BrdU, NeuN and NeuN/BrdU, and TH and TH/BrdU‐positive cells. The most optimal concentration (500 nmol/L) of APα significantly increased these positive cells of 6‐OHDA + DMSO group. In addition, Bic significantly decreased these double‐positive cells of 6‐OHDA + 500 nmol/L APα group (Figure 4F ~ I).

RETRACTED

### 3.7 APα treatment increased the phosphorylation of cytoplasmic CaMKIIδ3 and its nuclear translocation in 6‐OHDA‐lesioned mice

Since APα could open VGLCC in immature neurons,^8^, ^16^ we speculated that it might regulate the expression levels of Ca^2+^/CaM‐dependent protein kinases. Our morphological results demonstrated that CaMKIIδ3 was located in the multiple brain areas including the cerebral cortex, hippocampal dentate gyrus, SN, ventral tegmental area, LV‐, 3V‐, and Aq‐SVZ, and their surrounding regions (data not shown).

The relative expression levels of CaMKIIδ3 mRNA in the midbrain were much lower in 6‐OHDA + DMSO group than those in the normal saline + APα‐ or normal saline + Bic‐treated mice at 2 and 6 weeks following 6‐OHDA treatment. There was not significantly different among the normal saline + DMSO‐, normal saline + APα‐, and normal saline + Bic‐treated mice at 2 and 4 weeks following 6‐OHDA administration. As compared with 6‐OHDA + DMSO group, the relative expression levels of CaMKIIδ3 mRNA were significantly elevated after APα administration, and they were the highest on day 35 following APα administration. These effects were blocked by Bic treatment (Figure 5B).

**Figure 5:** (A), Representative protein bands for CaMKIIδ3 (55 kD) and p‐CaMKIIδ3 (80 kD) expression levels were shown in the cytoplasmic and nuclear fractions of midbrain. Lane 1 ~ 6: normal saline + DMSO, normal saline + APα, normal saline + Bic, 6‐OHDA + DMSO, 6‐OHDA + APα, and 6‐OHDA + APα+Bic groups at 2, 4, and 6 wk following 6‐OHDA injection; β‐actin (43 kD) or Histone H3 (17 kD): loading control. (B) and (C)~(F), Relative expression levels for CaMKIIδ3 mRNAs or CaMKIIδ3 and p‐CaMKIIδ3 proteins in the cytoplasmic and nuclear fractions of midbrain among groups. Values are mean ± SEM; n = 3 at various time points for each group. *P ＜ .05, **P ＜ .01, ***P ＜ .001, and ****P ＜ .0001, comparison between 6‐OHDA + DMSO and normal saline + DMSO or normal saline + APα or normal saline + Bic groups; ^#^ *P ＜ *.05, ^##^ *P ＜ *.01, ^###^ *P ＜ *.001, and ^####^ *P ＜ *.0001, comparison between 6‐OHDA + APα and 6‐OHDA + DMSO groups; ^&^ *P ＜ *.05, ^&&^ *P ＜ *.01, and ^&&&&^ *P ＜ *.0001, comparison between 6‐OHDA + APα+Bic and 6‐OHDA + APα groups; ^%^ *P ＜ *.05, comparison of CaMKIIδ3 mRNAs between normal saline + DMSO and normal saline + APα at 6 wk following 6‐OHDA injection; ^$^ *p＜*0.05, comparison of p‐CaMKIIδ3 expression levels between at 2 and 6 wk following 6‐OHDA injection in the cytoplasmic fraction of midbrain; ^^^ *P ＜ *.05, ^^^^^ *P ＜ *.001, and ^^^^^^ *P ＜ *.0001, comparison of CaMKIIδ3 mRNA or p‐CaMKIIδ3 protein expression levels between on day 7 or 21 and 35, as well as on day 7 and 21 or 35 following APα injection using *two‐way* ANOVA followed by Bonferroni post hoc test. NS, no significance

The effect of APα on total CaMKIIδ3 or p‐CaMKIIδ3 expression levels was further validated by Western blot assay (Figure 5A). The total CaMKIIδ3 or p‐CaMKIIδ3 expression levels in the midbrain were significantly decreased after 6‐OHDA treatment, as compared with normal saline + DMSO or normal saline + APα or normal saline + Bic groups. There was not significantly different among the normal saline + DMSO‐, normal saline + APα‐, and normal saline + Bic‐treated mice. Nevertheless, p‐CaMKIIδ3 expression levels were much higher in the cytoplasmic fraction of midbrain at 6 weeks than those at 2 and 4 weeks following 6‐OHDA injection. APα significantly increased the total CaMKIIδ3 or p‐CaMKIIδ3 expression levels on day 7 and 14 or 35 following APα administration, in particular, p‐CaMKIIδ3 expression levels were much higher in the cytoplasmic fraction of midbrain on day 21 and 35 than those on day 7 following APα administration. In addition, Bic significantly reduced the total CaMKIIδ3 or p‐CaMKIIδ3 expression levels on day 7 or 21 or 35 following APα administration (Figure 5C ~ F). Interestingly, our results showed that APα‐induced a ratio of p‐CaMKIIδ3/totalCaMKIIδ3 expression levels in the nuclear fraction was approximately 2.14‐fold higher than that in the cytoplasmic fraction of midbrain.

RETRACTED

### 3.8 APα treatment increased the expression levels of BDNF, CDK1, CDC2 or p‐CDC2 in the mRNAs or proteins of 6‐OHDA‐lesioned mice

The neurogenic action of APα predicted that it could regulate the neurotrophic factors and cell cycle proteins, so we examined the expression levels of BDNF and nuclear cyclin‐dependent kinase‐1 (CDK1) or cell division cycle protein 2 homolog (CDC2). Like CaMKIIδ3 mRNA expression levels, the relative expression levels of BDNF and CDC2 mRNAs in the midbrain were much lower in 6‐OHDA + DMSO group than those in normal saline + DMSO or normal saline + APα and normal saline + Bic groups at 2 and 4 weeks following 6‐OHDA treatment. There was not significantly different among the normal saline + DMSO‐, normal saline + APα‐, and normal saline + Bic‐treated mice. APα administration resulted in a significant upregulation, which was reversed by Bic administration (Figure 6A‐B). Western blot assay indicated that the protein expression levels of BDNF, CDK1, and p‐CDC2 had an entire consistence with their mRNAs expression levels at 2 or 4 or 6 weeks following 6‐OHDA treatment (Figure 6C,D ~ F).

**Figure 6:** (A) and (B), Relative level for BDNF (A) and CDC2 (B) mRNAs in the midbrain. (C) Representative protein bands for BDNF (28 kD), CDK1 (34 kD), and p‐CDC2 (34 kD) expression levels were shown in the midbrain. Lane 1 ~ 6: normal saline + DMSO, normal saline + APα, normal saline + Bic, 6‐OHDA + DMSO, 6‐OHDA + APα, and 6‐OHDA + APα+Bic groups at 2, 4, and 6 wk following 6‐OHDA injection; Histone H3 (17 kD): loading control. (D)~(F), BDNF (D), CDK1 (E), and p‐CDC2 (F) protein expression levels in the midbrain. Values are mean ± SEM; n = 3 at various time points for each group. *P ＜ .05, **P ＜ .01, ***P ＜ .001, and ****P ＜ .0001, comparison between 6‐OHDA + DMSO and normal saline + DMSO or normal saline + APα or normal saline + Bic groups; ^#^ *P ＜ *.05, ^##^ *P ＜ *.01, ^###^ *P ＜ *.001, and ^####^ *P ＜ *.0001, comparison between 6‐OHDA + APα and 6‐OHDA + DMSO groups; ^&^ *P ＜ *.05, ^&&^ *P ＜ *.01, ^&&&^ *P ＜ *.001, and ^&&&&^ *P ＜ *.0001, comparison between 6‐OHDA + APα+Bic and 6‐OHDA + APα groups using *two‐way* ANOVA followed by Bonferroni post hoc test. NS, no significance. (G) and (H), Co‐immunoprecipitation assay of total CaMKIIδ3/p‐CaMKIIδ and BDNF (G), as well as total CaMKIIδ3/p‐CaMKIIδ and CDK1 (H) interactions. Input: positive control; IgG: negative control; C: cytoplasmic fraction; N: nuclear fraction; IP: immunoprecipitation; IB: immunoblot; β‐actin (43 kD) or Histone H3 (17 kD): loading control

### 3.9 Co‐immunoprecipitation assay determined the interactions of CaMKIIδ3 or p‐CaMKIIδ3 and BDNF or CDK1

To determine the interaction of total CaMKIIδ3 or p‐CaMKIIδ3 with CDK1 or BDNF, co‐immunoprecipitation was performed. Our results demonstrated that a small fraction of CDK1 and BDNF were also present in the cytoplasmic fraction, although they were mainly located in the nuclear fraction of midbrain. Co‐immunoprecipitation assay revealed that total CaMKIIδ3and p‐CaMKIIδ3 predominantly bound to BDNF or CDK1 in the nuclear fraction of midbrain (Figure 6G‐H).

RETRACTED

## 4 DISCUSSION

Our current results indicated that 6‐OHDA‐induced reduction in TH‐positive fibers and the dopamine level terminally led to a massive loss of TH‐positive neurons, which was consistent with the previous reports.^26^, ^27^ Nevertheless, we also noticed there was a partial recovery at 6 weeks following 6‐OHDA injection including the striatal dopamine level or TH‐positive axon terminals, which seemed to be related to a substantial increase in X‐gal‐labeled Nestin‐positive NPCs at 4 weeks following 6‐OHDA injection by a postlesion compensatory mechanism. Although the neuronal death or degeneration could induce a modest increase in NPCs division or their neurogenesis,^28^, ^29^ their proliferation and differentiation could not keep up with the degenerative processes in an unfavorable microenvironment.^30^

In the aged and AD brains, a previous research has shown that there was a significant decrease in APα content, which was associated with a decrease in SNpc TH‐positive neurons.^10^, ^31^ Our current research further proved that APα treatment partly recovered the APα and dopamine levels in PD mice, which terminately protected the nigrostriatal TH‐positive neurons against 6‐OHDA lesion. Some studies indicated that APα regulated the neurogenesis of SVZ‐NPCs by binding to GABAAR and then opening L‐type Ca^2+^ channel.^14^, ^32^, ^33^ Once APα site within GABAAR was blocked by Bic, APα‐induced amelioration was abolished not only in SN‐striatal TH‐positive neurons but also in the proliferation and differentiation of newborn midbrain‐derived NPCs; however, Bic alone could not significantly decrease these indicators, suggesting that APα required GABAAR to promote the neurogenesis of NPCs.

GABAAR was a ligand‐gated chloride channel including a variety of subunits, and our results indicated that APα administration could significantly alleviate the expression levels of GABAAR α4 subunit in the membrane protein fraction of midbrain at 2 and 4 weeks following 6‐OHDA injection (*P* = .0244, *P* = .0022), which was significantly reversed on day 21 after pretreatment with Bic (*P* = .0447) (data not shown), but it did not suggest whether GABAARs was in a validated functional state. However, some studies reported that APa could induce a significant alteration in GABAAR expression levels by activating many GABAAR subtypes including GABAAα1 and GABAARβ2 in promoting the proliferation of NPCs, neuronal migration, synaptogenesis, and hippocampal neurogenesis.^14^, ^15^, ^18^

In the adult hippocampal neurogenesis, APα binding to GABAAR‐induced rise in the cytoplasmic Ca^2+^ concentration was often followed by the activation of gene transcription and intracellular cascades.^14^, ^18^, ^32^ Some studies reported that the cytoplasmic Ca^2+^/CaM activated and promoted the phosphorylation of CaMKII and its nuclear translocation, leading to the expressions of transcription factors and BDNF, which, in turn, promoted the neurite extension in 6‐OHDA‐lesioned dopaminergic neurons.^34^, ^35^ In CaMKII isoforms, our results indicated that CaMKIIδ3 was mainly located in the regions where NPCs were abundant except for SN and the striatum.^21^ As compared with the cytoplasmic fraction, APα could induce a higher ratio of p‐CaMKIIδ3/total CaMKIIδ3 in the nuclear fraction, indicating APα treatment enhanced the phosphorylation of cytoplasmic CaMKIIδ3 and its nuclear translocation in 6‐OHDA‐lesioned mice, which was in accordance with a previous report.^36^ However, a conflicting study indicated that p‐CaMKIIδ3 was dephosphorylated and then easily translocated into the nuclear fraction after the dopamine receptor was activated.^35^ This discrepancy might result from the idea that the assembly of CaMKII isoforms likely affected its activation and nuclear translocation.^37^

RETRACTED

Mohapel et al^38^ found that BDNF increased the number of newly formed cells in the striatum and SN of adult rats with a unilateral SN 6‐OHDA lesion. In the course of APα‐induced SVZ neurogenesis, BDNF phosphorylation was also elevated.^11^ In addition, APα could significantly upregulate the expression of proliferating cell nuclear antigen, cyclins, and CDKs.^39^, ^40^ Our studies demonstrated that APα increased CaMKIIδ3, BDNF, and CDC2 expression levels of 6‐OHDA‐lesioned mice via GABAAR by transcriptional and translational mechanisms. In addition, we also found that p‐CaMKIIδ3 or total CaMKIIδ3 had an interaction with CDK1 or BDNF, indicating that APα‐induced increase in the phosphorylation of cytoplasmic CaMKIIδ3 and its nuclear translocation further promoted their interactions with the cell cycle protein and BDNF, which, in turn, further increased these proteins expression levels.

Some studies and our previous results indicated that a small amount of SNpc newly generated TH‐positive neurons might be involved in the regeneration process of 6‐OHDA‐lesioned dopaminergic neurons.^9^, ^41^, ^42^, ^43^, ^44^ Our current results from the primarily cultured midbrain cells indicated that 6‐OHDA treatment could inhibit the acquisition of neuronal identities and reduce the newly generated midbrain‐derived NPCs differentiation toward mature neurons, which was not in line with Nestin‐positive NPCs in vivo study because a local unfavorable microenvironment could upregulate the number of Nestin‐positive NPCs with the absence of dopaminergic inputs.^9^ In addition, APα induced an extremely rare increase in the newborn dopaminergic neurons, which further supported that the newly formed NPCs and their differentiation contributed a small fraction to APα‐promoted regeneration process following 6‐OHDA lesion, indicating that the newborn mature neurons were formed after a strong selection of NPCs.^44^, ^45^

Some documents reported that APα increased the function of surviving dopaminergic neurons in a neighboring area to compensate the dysfunction from the lesioned neurons, which, in turn, enhanced the behavioral performance.^14^, ^15^, ^16^, ^46^ Other studies indicated that APα reinstated TH‐positive neurons and their fibers, as well as the motor symptoms in MPTP‐lesioned mice.^8^, ^17^, ^19^ Although there was a partial recovery in the turning behavior at 6 weeks following 6‐OHDA injection except for p‐CaMKIIδ3 expression, our results indicated that APα treatment could further improve the motor performance in PD mice, accompanying with a significant increase in TH‐positive neurons and their fibers or dopamine levels, as well as the number of NPCs. However, the detail mechanisms underlying APα‐ameliorated behavioral performance in 6‐OHDA‐lesioned mice need to be further elucidated.

RETRACTED

In conclusion, a vital contribution of the presented work is that APα/GABAAR/CaMKIIδ3 might be an alternative molecular and cellular mechanism that underlies APα‐treated PD.

## CONFLICT OF INTERESTS

The authors declare no conflict of interest.
